# High-Discrimination Comparison Algorithm for the Comprehensive Evaluation of Innovation Ability in Colleges and Universities under Uncertain Information

**DOI:** 10.1155/2022/7842651

**Published:** 2022-10-14

**Authors:** Ming Fu, Lifang Wang, Xueneng Cao, Bingyun Zheng, Xianxian Zhou, Shishu Yin

**Affiliations:** ^1^School of Management Science and Engineering, Anhui University of Finance & Economics, Bengbu 233030, Anhui, China; ^2^School of International Trade and Economics, Anhui University of Finance & Economics, Bengbu 233030, Anhui, China

## Abstract

The innovation ability of students is one of the most important objectives that need to be cultivated in colleges and universities. The comprehensive evaluation of innovation ability discussed in the study can be divided into two stages: the first stage can be called preliminary evaluation and its main target is to identify students with innovative potential; in the second stage, the target objects found in the previous stage will be evaluated quantitatively and ranked. However, it is always difficult to quantitatively evaluate the innovation ability by using traditional algorithms. Based on the above analysis, the study proposes an algorithm to quantitatively evaluate the innovation ability with the help of management thought and fuzzy mathematics. Data are the basis of evaluation, and the accuracy of the data directly determines the quality of the algorithm; the data structure of the incompletely probabilistic fuzzy set is proposed in the study; the data structure can fully consider the fuzziness of the problem and the hesitation in the decision-making process; it can save the original detailed data to the maximum extent. Certainly, certain information may be lost or only the value range can be determined; there are usually some unknowns in the evaluation data, and the consistency optimization model is proposed for solving the problem. Usually, there are certain contradictions among the evaluation data; the definition of the consistency degree is proposed in the study; the consistency can be verified in time after all the unknowns are obtained, and the automatic adjustment module will be activated immediately if the value of the consistency degree exceeds the warning threshold. Finally, after verifying the data consistency, the solution can be obtained by solving the optimization model. Several experiments have been carried out to verify the effectiveness and high-discrimination ability of the algorithm proposed in the study; meanwhile, the superiority of the algorithm is further verified through comparisons with other outstanding algorithms.

## 1. Introduction

Innovation ability has always been an important force to promote human progress which has been recognized by more and more experts. The innovation ability of students is one of the training targets of higher education; it is also one of the core indicators to measure the quality of education. However, the quantitative measurement of the innovation ability is seriously insufficient currently.

Innovation is a kind of human creative practice from the perspective of philosophy; innovation is the activity that people discover or produce some novel, unique, valuable new products and new ideas in order to meet the needs of development from the perspective of sociology. Innovation is the behavior of creating new inventions and obtaining certain beneficial effects by using existing knowledge and materials from the perspective of economics. From the above analysis, we can see that no matter from which perspective, innovation is a relatively vague and subjective concept.

At present, academic circles have generally believed that innovation ability is composed of numerous factors, but its specific structure is still an unsolved problem. The existing research studies on the structure of innovation ability are mainly based on personality theory, competency theory, and action theory. The personality theory holds that innovative behavior is closely related to creative personality, risk-taking spirit, and self-efficacy; on the basis of the personality theory, the competency theory mainly focuses on the combination method of personality and behavior; the action theory believes that the essence of innovation is action, and it provides theoretical support for exploring the internal logic contained in the innovation ability structure. Generally, the theoretical discussions on the innovation ability have provided important academic accumulation for this study; however, there are also shortcomings, the fault tolerance of the model is relatively low, and the accuracy of the results needs to be further improved.

Professor Zadeh first put forward the concept of fuzzy sets in 1965 [1], the emergence of fuzzy sets makes it possible to deal with fuzzy problems by mathematical methods, its core idea is to extend the characteristic function to a value in the closed interval [0, 1], and the value is used to describe the fuzzy degree of the element in a set. This idea was widely recognized by scholars, and since then, the fuzzy sets have developed rapidly and expanded into many forms, including L-type fuzzy sets, 2-type fuzzy sets, interval fuzzy sets, hesitation fuzzy sets, probability hesitation fuzzy sets, hesitation fuzzy linguistic sets, and probability hesitation fuzzy linguistic sets. The definition of the L-type fuzzy sets was proposed by Goguen in 1967 [2], different from fuzzy sets; it expands the value range of membership function into a partially ordered set. The 2-type fuzzy sets which allow membership to be a fuzzy set can be regarded as a special case of the L-type fuzzy sets. The interval fuzzy sets allow the membership to be interval values. The three fuzzy sets discussed above only consider the value of membership function; they cannot describe the information of support, opposition, and hesitation simultaneously in practical applications; moreover, due to the complexity of problems, people are often hesitant and difficult to reach consensuses in the process of collaborative decision-making and evaluation, and the data collected may be positive, negative, and hesitant; therefore, the Bulgarian scholar Atanassov extended the definition of the fuzzy set and successively proposed the concepts of intuitionistic fuzzy sets and interval intuitionistic fuzzy sets [3], and the membership, nonmembership, and hesitation can be considered simultaneously. Torra, a Spanish scholar, further expanded the fuzzy sets and proposed the definition of the hesitation fuzzy sets in 2010 [4]; when evaluating alternatives, people often hesitate among multiple values; therefore, ordinary data structures are difficult to handle this problem; fortunately, the hesitation fuzzy set can effectively solve this problem by saving all the possible values; it can be seen that the hesitant fuzzy set can more accurately and reasonably describe the uncertainty of objects; therefore, it is widely used in dealing with fuzzy problems. We find that the hesitant fuzzy set cannot directly reflect the number of experts in the group decision-making and a lot of information may be lost. Based on the above considerations, scholars proposed the definition of the probability hesitation fuzzy set which is an extension of the hesitation fuzzy set, and its basic element is composed of the evaluation value and its corresponding probability; the probability can accurately describe the importance or occurrence rate of the evaluation value. Usually, verbal words rather than mathematical symbols are more commonly used to describe evaluation opinions in real life; this is obviously beyond the capability of hesitant fuzzy sets, and for this reason, Rodriguez proposed the definition of hesitant fuzzy linguistic sets [5].

Obviously, people are better at making pairwise comparisons between alternatives in the process of decision-making; it is always easier to obtain reasonable results by pairwise comparisons; the preference relationship table which records all comparison results will be obtained after multiple pairwise comparisons. In order to describe the relative importance of comparison results, Saaty proposed the definition of the fundamental scale [6]; while each element in the fundamental scale is in the form of a single real-value, due to the complexity and uncertainty of decision-making problems and the incompleteness of information or knowledge, it is often difficult to obtain these exact values; therefore, Maji et al. used fuzzy membership functions to describe the relative importance of comparison results [7]; unfortunately, the preference relationship established by the method of Maji does not satisfy the complementary condition; in order to solve this problem, Soller et al. proposed the method of the fuzzy preference relation which can effectively overcome this defect [8]; moreover, there are inevitable contradictions among the data in the preference relationship table; the definition of the consistency is introduced to describe the contradiction degree and it is one of important concepts in the preference relationship theory; the solutions that do not satisfy consistency requirement are not feasible. Stukalina proposed a calculation method of priority weights that satisfies the consistency preference relationship [9]. Xu defined the consistency of intuitionistic fuzzy preference relationship [10].

At present, the comprehensive evaluation of innovation ability in colleges and universities is indeed a worthy problem for studying; it has not only certain theoretical value but also practical value; however, innovation ability is a vague and subjective concept, which is difficult to measure scientifically and accurately; some key indicators of the problem are often difficult to be described by single determined values; even worse, due to the limitation of cognition and the complexity of the problem, some information may be lost; therefore, traditional algorithms are hard to deal with this problem. The study combines the problem with the fuzzy theory and provides a new way to solve this problem from the perspective of management science.

## 2. Some Basic Definitions and Theories

Some basic definitions and theories will be briefly introduced in this section which will be helpful for other researchers to better understand the algorithm proposed in this study.

### 2.1. The Incompletely Probabilistic Fuzzy Set

The definition of the incompletely probabilistic fuzzy set (IPFS) is expanded from the interval-valued fuzzy set and the probability hesitation fuzzy set, which can be described mathematically as follows:

(1) $$\begin{array}{c} l_{rs}=\left\{\gamma_{l}|p_{l}\;\gamma_{l}\in \left[0,1\right],p_{l}\in \left[0,1\right],\overset{k}{\underset{l=1}{\sum }}p_{l}=1,l=1,2,\cdots ,k\right\}. \end{array}$$

The symbol *γ*_*l*_ indicates one of the evaluation values, the symbol *p*_*l*_ indicates the corresponding probability value of the evaluation value *γ*_*l*_, the restriction *p*_*l*_ ∈ [0,1] indicates the value range of the evaluation value *γ*_*l*_, and the restriction ∑_*l*=1_^*m*^*p*_*l*_=1 indicates that the sum of all the probability values must be equal to 1. In general, any incompletely probabilistic fuzzy set *l*_*rs*_ can include several elements, the total number of elements is recorded as the symbol *k*, each pair of the symbols *γ*_*l*_*|p*_*l*_ can be called the incompletely probabilistic fuzzy element (IPFE), and the restriction *l*=1,2, ⋯, *k* can be regarded as the value range of subscripts.

Different from other data structures, multiple values can be stored together in a single incompletely probabilistic fuzzy set, which can overcome hesitation in the evaluation process; in addition, the probability values can provide additional descriptions for the evaluation values; furthermore, it is worth noting that the evaluation values and the probability values are allowed to contain some unknowns; this improvement will further expand the application scope.

Let us illustrate the above theory with several simple examples. It can be divided into several categories according to the unknowns: the first category is that all the information is known, such as *l*_12_={0.32*|*0.42,0.38|0.26,0.42|0.32}; the second category is that some evaluation information is unknown, such as *l*_13_={*x*_1_*|*0.42,0.38|0.26,0.42|0.32}; the third category is that some probability information is unknown, such as *l*_14_={0.32*|*0.42,0.38|*y*_1_, 0.42|(0.58 − *y*_1_)} and *l*_23_={0.32*|y*_2_, 0.38|*y*_3_, 0.42|(1 − *y*_2_ − *y*_3_)}; the fourth category is that some evaluation information and probability information are unknown, such as *l*_24_={0.32*|y*_3_, *x*_2_|(1 − *y*_3_ − *y*_4_), 0.42|*y*_4_}. We must point out that the default value range of unknowns is from 0 to 1; however, if possible, it is still recommended to give the value ranges of unknowns, which can improve the accuracy of the algorithm.

Through the above analysis, we find that the data structure proposed in the paper can save the original data to the greatest extent. In addition, the expected value of the incompletely probabilistic fuzzy set may be used in the latter subsections, and the definition of the expected value is shown as follows:

(2) $$\begin{array}{c} E\left(l_{rs}\right)=\overset{k}{\underset{l=1}{\sum }}\gamma_{l}\cdot p_{l}\text{.} \end{array}$$

The expected values of the above incompletely probabilistic fuzzy sets can be calculated according to equation (2) and are shown as follows:

(3) $$\begin{array}{c} E\left(l_{12}\right)=E\left(\left\{0.32|0.42,0.38\left|0.26,0.42\right|0.32\right\}\right)=0.3676\text{,}\\ E\left(l_{13}\right)=E\left(\left\{x_{1}|0.42,0.38\left|0.26,0.42\right|0.32\right\}\right)=0.2332+0.42\cdot x_{1}\text{,}\\ E\left(l_{14}\right)=E\left(\left\{0.32|0.42,0.38\left|y_{1},0.42\right|\left(0.58-y_{1}\right)\right\}\right)=0.378-0.04\cdot y_{1}\text{.} \end{array}$$

(4) $$\begin{array}{c} E\left(l_{23}\right)=E\left(\left\{0.32|y_{2},0.38\left|y_{3},0.42\right|\left(1-y_{2}-y_{3}\right)\right\}\right)=0.42-0.1\cdot y_{2}-0.04\cdot y_{3}\text{,}\\ E\left(l_{24}\right)=E\left(\left\{0.32|y_{3},x_{2}\left|\left(1-y_{3}-y_{4}\right),0.42\right|y_{4}\right\}\right)=\left(0.32-x_{2}\right)\cdot y_{3}+x_{2}+\left(0.42-x_{2}\right)\cdot y_{4}\text{.} \end{array}$$

### 2.2. The Subtraction of Incompletely Probabilistic Fuzzy Sets

The subtraction of incompletely probabilistic fuzzy sets should be used in the following sections; however, since the definition of the incompletely probabilistic fuzzy set is first proposed in the paper, this method is rarely mentioned by other researchers; therefore, it is necessary to define the subtraction of incompletely probabilistic fuzzy sets which is shown as follows:

(5) $$\begin{array}{c} l_{xy}=\left\{\gamma_{l_{1}}|p_{l_{1}}\;\gamma_{l_{1}}\in \left[0,1\right],p_{l_{1}}\in \left[0,1\right],\overset{k_{1}}{\underset{l_{1}=1}{\sum }}p_{l_{1}}=1,l_{1}=1,2,\cdots ,k_{1}\right\}\text{,}\\ l_{pq}=\left\{\gamma_{l_{2}}|p_{l_{2}}\;\gamma_{l_{2}}\in \left[0,1\right],p_{l_{2}}\in \left[0,1\right],\overset{k_{2}}{\underset{l_{2}=1}{\sum }}p_{l_{2}}=1,l_{2}=1,2,\cdots ,k_{2}\right\}\text{,}\\ l_{\mathrm{\#x394;}}=l_{xy}-l_{pq}=\underset{\gamma_{l_{1}}\in l_{xy},\gamma_{l_{2}}\in l_{pq},p_{l_{1}}\in l_{xy},p_{l_{2}}\in l_{pq}}{\cup }\left\{\left(\gamma_{l_{1}}-\gamma_{l_{12}}\right)|p_{l_{1}}\cdot p_{l_{2}}\;l_{1}=1,2,\cdots ,k_{1},l_{2}=1,2,\cdots ,k_{2}\right\}\text{.} \end{array}$$

The symbols *l*_*xy*_ and *l*_*pq*_ represent two ordinary *IPFS*_*s*_, and the symbol *l*_Δ_ records the subtraction result of the two ordinary *IPFS*_*s*_. In particular, as a special case, the complementary set of the incompletely probabilistic fuzzy set will be frequently used in later sections; therefore, the definition of the complementary set can be given in advance which is shown as follows:

(6) $$\begin{array}{c} l_{rs}^{c}=1-l_{rs}=\left\{\left(1-\gamma_{l}\right)|p_{l}\;\gamma_{l}\in \left[0,1\right],p_{l}\in \left[0,1\right],\overset{k}{\underset{l=1}{\sum }}p_{l}=1,l=1,2,\cdots ,k\right\}. \end{array}$$

Let us give a few simple examples to illustrate the above theory; the values of the *l*_12_, *l*_13_, *l*_14_, *l*_23_, *l*_24_ have been given in the above subsection, and the specific calculation steps of the complementary sets are shown as follows:

(7) $$\begin{array}{c} l_{12}^{c}=1-l_{12}=1-\left\{0.32|0.42,0.38\left|0.26,0.42\right|0.32\right\}=\left\{0.68|0.42,0.62\left|0.26,0.58\right|0.32\right\}\text{,}\\ l_{13}^{c}=1-l_{13}=1-\left\{x_{1}|0.42,0.38\left|0.26,0.42\right|0.32\right\}=\left\{\left(1-x_{1}\right)|0.42,0.62\left|0.26,0.58\right|0.32\right\}\text{,}\\ l_{14}^{c}=1-l_{14}=1-\left\{0.32|0.42,0.38\left|y_{1},0.42\right|0.58-y_{1}\right\}=\left\{0.68|0.42,0.62\left|y_{1},0.58\right|\left(0.58-y_{1}\right)\right\}\text{,} \end{array}$$

(8) $$\begin{array}{c} l_{23}^{c}=1-l_{23}=1-\left\{0.32|y_{2},0.38\left|y_{3},0.42\right|\left(1-y_{2}-y_{3}\right)\right\}=\left\{0.68|y_{2},0.62\left|y_{3},0.58\right|\left(1-y_{2}-y_{3}\right)\right\}\text{,}\\ l_{24}^{c}=1-l_{24}=1-\left\{0.32|y_{3},x_{2}\left|\left(1-y_{3}-y_{4}\right),0.42\right|y_{4}\right\}=\left\{0.68|y_{3},\left(1-x_{2}\right)\left|\left(1-y_{3}-y_{4}\right),0.58\right|y_{4}\right\}\text{.} \end{array}$$

### 2.3. The Comparison Decision-Making Method

The goal of decision-making can be simply summarized as finding the best solution from multiple alternatives [11]. Specifically, the goal of this paper is to rank students according to the innovation ability. With the help of management science, every student with innovative potential can be regarded as an alternative.

All the alternatives can be recorded as mathematically. Data are always the basis of any decision-making [12]; first, several indicators will be selected from multiple interference factors which can be recorded as *I*={*I*_1_, *I*_2_,…, *I*_*t*_}, the data of each indicator needs to be collected and recorded, and the data structure of the incompletely probabilistic fuzzy set mentioned above is suitable for collecting the original information. All the indicators can be classified into two categories according to the objective function: positive indicators and negative indicators. The negative indicators should be converted into positive indicators by using the complement operation mentioned in equation (3). The overall structure of the original data needs to be collected is listed in Table 1.

Generally, the alternatives can be ranked based on the data in the above table when the data are complete; unfortunately, due to the fuzziness of the problem and the hesitation of experts [13], the data in the table often contain several unknowns which will directly make the problem cannot be solved by common algorithms; for this reason, the comparison decision-making algorithm based on the incompletely probabilistic fuzzy set is proposed in the paper.

Compared with multiple alternatives, when only two alternatives are compared at a time, it is obvious that people can give the evaluation result with higher accuracy [14]. Based on this idea, the comparison table of alternatives can be created, and the structure of the comparison table is shown as Table 2.

Every element *l*_*ij*_ in Table 2 is in the form of the incompletely probabilistic fuzzy set. The elements in the above table meet the following two rules: the first one is that all the elements in the main diagonal should be recorded as {0.5*|*1} which can be denoted as *l*_*ii*_={0.5*|*1}∀ *i*=1,2, ⋯, *m* completely; obviously, it is the inevitable result when compared with themselves; the other rule is that the elements symmetrical to the main diagonal will meet complementary relationship which can be denoted as *l*_*ij*_=*l*_*ji*_^*c*^∀ *i*, *j*=1,2, ⋯, *m* mathematically. After the above analysis, we can find that only the elements on the upper triangle of Table 3 need to be evaluated, and the data in Table 1 can play an important role in this process [15].

### 2.4. The Consistency Problem in the Process of Group Decision-Making

Every data in Table 3 is obtained separately by comparing only two alternatives at one time; all alternatives have never been compared together; therefore, there may be some inconsistencies among the data.

Inspired by Herrera [16], we believe that the data in Table 3 will meet the consistency requirement if equation (5) holds.

(9) $$\begin{array}{c} E\left(l_{rs}\right)=E\left(l_{rk}\right)-E\left(l_{sk}\right)+0.5\forall r,s,k=1,2,\cdots ,m. \end{array}$$

While, how to make equation (5) hold has become a difficult problem in front of us. Based on the theory of Chiclana et al. [17], the data *C*=(*l*_*ij*_)_*m*×*m*_ will meet the consistency requirement if and only if there is a set of normalized values *ω*=(*ω*_1_, *ω*_2_, ⋯,*ω*_*m*_)^*T*^ that make the following equations hold [18]:

(10) $$\begin{array}{c} E\left(l_{rs}\right)=In\omega_{r}-In\omega_{s}+0.5\forall r,s=1,2,\cdots m. \end{array}$$

The symbol *ω*_*i*_ can also be called the comprehensive value of the alternative *A*_*i*_. Generally, it can be calculated by the following equation:

(11) $$\begin{array}{c} \omega_{r}=\frac{e^{1/m\overset{m}{\underset{k=1}{\sum }}E\left(l_{rk}\right)}}{\overset{m}{\underset{j=1}{\sum }}e^{1/m\overset{m}{\underset{k=1}{\sum }}E\left(l_{jk}\right)}}\forall r,j,k=1,2,\cdots ,m. \end{array}$$

According to formula (6), the proof of the necessary condition is shown as follows:

(12) $$\begin{array}{c} In\omega_{r}-In\omega_{s}=\frac{1}{m}\overset{m}{\underset{k=1}{\sum }}E\left(l_{rk}\right)-\frac{1}{m}\overset{m}{\underset{k=1}{\sum }}E\left(l_{sk}\right)=\frac{1}{m}\overset{m}{\underset{k=1}{\sum }}\left(E\left(l_{rk}\right)-E\left(l_{sk}\right)\right)=\frac{1}{m}\overset{m}{\underset{k=1}{\sum }}\left(E\left(l_{rs}\right)-0.5\right)=\frac{1}{m}\times m\times \left(E\left(l_{rs}\right)-0.5\right)=E\left(l_{rs}\right)-0.5\text{.} \end{array}$$

Thus, the equation *E*(*l*_*rs*_)=*Inω*_*r*_ − *Inω*_*s*_+0.5 can be derived from the positive direction [19]. Conversely, the proof of the sufficient condition is shown as follows:

(13) $$\begin{array}{c} \begin{array}{c} E\left(l_{rs}\right)=In\omega_{r}-In\omega_{s}+0.5\\ =\left(In\omega_{r}-In\omega_{k}+0.5\right)-\left(In\omega_{s}-In\omega_{k}+0.5\right)+0.5\\ =E\left(l_{rk}\right)-E\left(l_{sk}\right)+0.5\text{.} \end{array}\text{.} \end{array}$$

Thus, the equation *E*(*l*_*rs*_)=*E*(*l*_*rk*_) − *E*(*l*_*sk*_)+0.5 can be derived from the opposite direction. In addition, when the equation *E*(*l*_*rs*_)=∑_*l*=1_^*k*^*γ*_*l*_ · *p*_*l*_=*Inω*_*r*_ − *Inω*_*s*_+0.5 holds, then equation (7) will also hold [20], and the derivation process is shown as follows:

(14) $$\begin{array}{c} E\left(l_{sr}\right)=In\omega_{s}-In\omega_{r}+0.5\text{,} \end{array}$$

(15) $$\begin{array}{c} E\left(l_{sr}\right)=E\left(l_{rs}^{c}\right)=E\left(1-l_{rs}\right)\\ =\overset{k}{\underset{l=1}{\sum }}p_{l}-\overset{k}{\underset{l=1}{\sum }}\gamma_{l}\cdot p_{l}\\ =1-\left(In\omega_{r}-In\omega_{s}+0.5\right)\\ =In\omega_{s}-In\omega_{r}+0.5\text{.} \end{array}$$

Therefore, according to the above analysis, it is only necessary to verify the consistency of the upper triangle data in Table 3.

## 3. The High-Discrimination Comparison Algorithm

The algorithm proposed in this paper mainly focuses on the alternatives with small differences and is difficult to be ranked directly; the algorithm and the mathematical model will be systematically introduced in this section. The flowchart of the high-discrimination comparison algorithm is shown in Figure 1.

### 3.1. Mathematicise the Problem

First, list all the alternatives that need to be ranked and divide them into two categories: the first category is the alternatives that can be ranked directly by common methods and the other category is the alternatives that are difficult to be ranked and need the help of the algorithm proposed in the paper [21]; these alternatives can be recorded as *A*={*A*_1_, *A*_2_, ⋯, *A*_*m*_}.

After that, several key indicators will be selected and can be denoted as *I*={*I*_1_, *I*_2_, ⋯, *I*_*t*_}; the original data of each indicator will be collected and then standardized; then, the processed data *I*=(*l*_*ij*_)_*m*×*t*_∀ *i*=1,2, ⋯, *m*; *j*=1,2, ⋯, *t* will be saved in the form of the incompletely probabilistic fuzzy set.

The comparison table will be established through multiple pairwise comparisons among different alternatives. The values in the comparison table can be obtained mainly based on the key indicators of the alternatives mentioned in the above step. The data of the comparison table can be denoted as *C*=(*l*_*ij*_)_*m*×*m*_∀ *i*, *j*=1,2, ⋯, *m*. Since all the alternatives have not been compared together, there may be some contradictions among the data in the comparison table [22], and we must point out that the data cannot be used for ranking alternatives until it meets the requirement of consistency verification. The consistency optimization model and the adjustment algorithm will be introduced in detail in the following subsections.

### 3.2. The Consistency Optimization Model

Due to the complementary relationship mentioned above, the consistency optimization model is proposed according to the elements in the upper triangle of the comparison table. The consistency constraints can be established by introducing positive deviations and negative deviations [23]; the objective function is to minimize the sum of deviations. The model is shown as follows:

(16) $$\begin{array}{c} \begin{array}{c} Mo\;de\;l\;1\text{:}\\ \min\;\xi =\min\overset{m-1}{\underset{i=1}{\sum }}\overset{m}{\underset{j>i}{\sum }}\left(d_{ij}^{+}+d_{ij}^{-}\right),\\ s.t.\left\{\begin{array}{c} In\omega_{i}-In\omega_{j}+0.5-\overset{k}{\underset{l=1}{\sum }}\gamma_{l}\cdot p_{l}-d_{ij}^{+}+d_{ij}^{-}=0\\ \overset{m}{\underset{i=1}{\sum }}\omega_{i}=1\\ 0\leq \omega_{i}\leq 1\\ 0\leq d_{ij}^{+}\leq 1\\ 0\leq d_{ij}^{-}\leq 1\\ i=1,2,\cdots ,m\\ j=1,2,\cdots ,m\\ i<j \end{array}\right. \end{array}\text{.} \end{array}$$

Although the accuracy of each comparison result obtained by such a method is relatively high from the local perspective, however, as mentioned above, only two alternatives are compared at a time, and the data may be inconsistent from the whole perspective [24]. For this reason, we propose the definition of the consistency degree which is shown as follows:

(17) $$\begin{array}{c} CI=\frac{2}{m\left(m-1\right)}\overset{m-1}{\underset{i=1}{\sum }}\overset{m}{\underset{j>i}{\sum }}\left(d_{ij}^{+}+d_{ij}^{-}\right). \end{array}$$

The consistency threshold (Ω) will be set in advance, if the inequality *CI* ≤ Ω holds, which indicates that the data meet the consistency requirement, and the calculation results obtained by the model 1 will be valid [25]; on the other hand, if the inequality *CI* > Ω holds, it indicates that some data in the comparison table must be adjusted in time, and the specific method will be introduced in the next subsection.

### 3.3. The Consistency Automatic Adjustment Algorithm

The flowchart of the consistency automatic adjustment algorithm is shown in Figure 2. The adjustment method can be divided into several steps, which are introduced in detail as follows:

1. Find the maximum deviation value which can be described as *d*_max_=max {*d*_*ij*_^+^, *d*_*ij*_^−^*|*∀ *i*, *j*=1,2, ⋯, *m*; *i* < *j*} mathematically
2. It can be divided into two categories according to whether the maximum deviation is positive or negative [26]. If the value is positive which can be denoted as *d*_max_=*d*_*ij*_^+^, then find the maximum probability value in the corresponding incompletely probabilistic fuzzy set *l*_*ij*_ which can be denoted as *p*_*ij*,*l*_^max^, and the corresponding evaluation value *r*_*ij*,*l*_ will increase *d*_max_ which can be described as *r*_*ij*,*l*_=*r*_*ij*,*l*_+*d*_max_ mathematically; similarly, if the value is negative which can be denoted as *d*_max_=*d*_*ij*_^−^, then find the maximum probability value in the corresponding incompletely probabilistic fuzzy set *l*_*ij*_ which can be denoted as *p*_*ij*,*l*_^max^, and the corresponding evaluation value *r*_*ij*,*l*_ will decrease *d*_max_, which can be described as *r*_*ij*,*l*_=*r*_*ij*,*l*_ − *d*_max_ mathematically.
3. The consistency verification operations listed in the previous subsection will be executed repeatedly until the consistency requirement is met
4. Finally, the alternatives will be ranked according to the values of *ω*_*i*_(*i*=1,2, ⋯, *m*)

## 4. A Case of the Comparison Algorithm Based on Uncertain Information

### 4.1. The General Description of the Problem

Innovation ability is the soul of national progress and the core of economic competition [27]. As the main institutions for cultivating innovative talents, universities or colleges have always attached great importance to the cultivation of innovation ability. Finding students with innovative potential as soon as possible is very important for the work of cultivating innovative talents; however, innovation ability is a vague concept and difficult to be measured quantitatively [28]. Based on these analyses, the algorithm proposed in this paper is suitable for dealing with such problems.

Supposing, after the first round of screening, four students with innovative potential are found out, and we hope to rank them according to their innovative ability. The four students can be denoted as {*A*_1_, *A*_2_, *A*_3_, *A*_4_}. Comparisons will be made between any two students, and the results given by experts will be recorded in the form of incompletely probabilistic fuzzy sets; thus, the comparison table will be established, and the consistency threshold is set as Ω=0.015.

According to the comparison data, it can be divided into several categories, which will be introduced, respectively, in the following subsections.

### 4.2. The Comparison Algorithm with Complete Information

In this category, all the data are complete, such as the data in Table 4. Due to the complementary relationship mentioned above, the elements in the lower triangle are not listed for the sake of simplicity, and the elements in the upper triangle and the main diagonal are given.

We find that it is almost impossible to rank the alternatives directly based on the data in the above table, the optimization model mentioned above will be built and its extended form is shown as follows:

(18) $$\begin{array}{c} Mo\;de\;l\;2\text{:}\\ \min\xi_{1}=d_{12}^{+}+d_{12}^{-}+d_{13}^{+}+d_{13}^{-}+d_{14}^{+}+d_{14}^{-}+d_{23}^{+}+d_{23}^{-}+d_{24}^{+}+d_{24}^{-}+d_{34}^{+}+d_{34}^{-}\\ s.t.\left\{\begin{array}{c} In\omega_{1}-In\omega_{2}+0.5-0.4786-d_{12}^{+}+d_{12}^{-}=0\\ In\omega_{1}-In\omega_{3}+0.5-0.4894-d_{13}^{+}+d_{13}^{-}=0\\ In\omega_{1}-In\omega_{4}+0.5-0.5431-d_{14}^{+}+d_{14}^{-}=0\\ In\omega_{2}-In\omega_{3}+0.5-0.5288-d_{23}^{+}+d_{23}^{-}=0\\ In\omega_{2}-In\omega_{4}+0.5-0.4743-d_{24}^{+}+d_{24}^{-}=0\\ In\omega_{3}-In\omega_{4}+0.5-0.5356-d_{34}^{+}+d_{34}^{-}=0\\ \overset{4}{\underset{r=1}{\sum }}\omega_{i}=1\\ 0\leq \omega_{i}\leq 1,\;i=1,2,3,4\\ 0\leq d_{jk}\leq 1,\;j=1,2,3,\;k=2,3,4 \end{array}\right.\text{.} \end{array}$$

The above linear model can be solved with the help of the lingo software, and the calculation results are shown as follows:

(19) $$\begin{array}{c} \xi_{1}=0.1082\text{,}\\ d_{13}^{+}=0.00905;d_{14}^{-}=0.00905;d_{23}^{-}=0.00895;d_{24}^{+}=0.08115\text{,} \end{array}$$

(20) $$\begin{array}{c} d_{12}^{+}=d_{12}^{-}=d_{13}^{-}=d_{14}^{+}=d_{23}^{+}=d_{24}^{-}=d_{34}^{+}=d_{34}^{-}=0. \end{array}$$

The value of the consistency degree *CI* can be calculated according to equation (8); the value is *CI*=0.018 after calculation. We can find that the inequality *CI* ≤ Ω does not hold, and the data in Table 4 do not pass the consistency verification, which indicates that the reliability of the results is not enough; consequently, the consistency adjustment module will be activated immediately; the specific steps are listed as follows:

(1) The maximum deviation is found which is denoted as *d*_max_=max {*d*_*ij*_^+^, *d*_*ij*_^−^}=*d*_24_^+^, and its type is a positive deviation.
(2) We can find that the evaluation value of the *l*_24_ is denoted as *l*_24_=(0.46*|*0.44,0.48|0.25,0.49|0.31) in the above table. The maximum probability value in the *l*_24_ is 0.44; therefore, the corresponding evaluation value will be increased from 0.46 to 0.54115, and the specific calculation step is *r*_*ij*,*l*_=*r*_*ij*,*l*_+*d*_max_=0.46+0.08115=0.54115 according to the above adjustment algorithm. So, the updated value of the *l*_24_′ will be denoted as *l*_24_′=(0.54115*|*0.44,0.48|0.25,0.49|0.31) after the first adjustment.
(3) The model will be rebuilt based on the updated data, and it is shown as follows:
  (21) $$\begin{array}{c} Mo\;de\;l\;3:\min\xi_{1}^{\prime }={d_{12}^{+}}^{\prime }{\;}^{+}{d_{12}^{-}}^{\prime }+{d_{13}^{+}}^{\prime }+{d_{13}^{-}}^{\prime }+{d_{14}^{+}}^{\prime }+{d_{14}^{-}}^{\prime }+{d_{23}^{+}}^{\prime }+{d_{23}^{-}}^{\prime }+{d_{24}^{+}}^{\prime }+{d_{24}^{-}}^{\prime }+{d_{34}^{+}}^{\prime }+{d_{34}^{-}}^{\prime }\\ s.t.\left\{\begin{array}{c} In\omega_{1}^{\prime }-In\omega_{2}^{\prime }+0.5-0.4786-{d_{12}^{+}}^{\prime }+{d_{12}^{-}}^{\prime }=0\\ In\omega_{1}^{\prime }-In\omega_{3}^{\prime }+0.5-0.4894-{d_{13}^{+}}^{\prime }+{d_{13}^{-}}^{\prime }=0\\ In\omega_{1}^{\prime }-In\omega_{4}^{\prime }+0.5-0.5431-{d_{14}^{+}}^{\prime }+{d_{14}^{-}}^{\prime }=0\\ In\omega_{2}^{\prime }-In\omega_{3}^{\prime }+0.5-0.5288-{d_{23}^{+}}^{\prime }+{d_{23}^{-}}^{\prime }=0\\ In\omega_{2}^{\prime }-In\omega_{4}^{\prime }+0.5-0.510006-{d_{24}^{+}}^{\prime }+{d_{24}^{-}}^{\prime }=0\\ In\omega_{3}^{\prime }-In\omega_{4}^{\prime }+0.5-0.5356-{d_{34}^{+}}^{\prime }+{d_{34}^{-}}^{\prime }=0\\ \overset{4}{\underset{r=1}{\sum }}\omega_{i}^{\prime }=1\\ 0\leq \omega_{i}^{\prime }\leq 1,\;i=1,2,3,4\\ 0\leq d_{jk}^{\prime }\leq 1,\;j=1,2,3,\;k=2,3,4 \end{array}\right.\text{.} \end{array}$$

The model can be solved again with the help of the lingo software and the results are shown as follows: *ξ*_1_′=0.072494;

(22) $$\begin{array}{c} \omega_{1}^{\prime }=0.2506452;\omega_{2}^{\prime }=0.2560668;\omega_{3}^{\prime }=0.2510339;\omega_{4}^{\prime }=0.2422541\text{,}\\ {d_{13}^{+}}^{\prime }=0.00905;{d_{14}^{-}}^{\prime }=0.00905;{d_{23}^{-}}^{\prime }=0.00895;{d_{24}^{+}}^{\prime }=0.045444\text{,}\\ {d_{12}^{+}}^{\prime }={d_{12}^{-}}^{\prime }={d_{13}^{-}}^{\prime }={d_{14}^{+}}^{\prime }={d_{23}^{+}}^{\prime }={d_{24}^{-}}^{\prime }={d_{34}^{+}}^{\prime }={d_{34}^{-}}^{\prime }=0\text{.} \end{array}$$

The value of the consistency degree *CI* can be calculated according to equation (8), and the value is *CI*′=0.01208 after calculation. We can find that the inequality *ξ*_1_′ < Ω holds after the adjustment which indicates that the calculation results meet the consistency requirements; therefore, the result is reasonable, and it is *A*_2_≻*A*_3_≻*A*_1_≻*A*_4_ according to the innovative ability.

### 4.3. The Comparison Algorithm with Unrelated Unknowns

In this category, the data contain several unknowns and the unknowns are not related to each other, such as the data in Table 5. Each unknown may give a specific value range; if it is not given, the default value range of the unknown is 0 ≤ *x* ≤ 1.


(23) $$\begin{array}{c} 0.50\leq x_{1}\leq 0.54;0.48\leq x_{2}\leq 0.52;0.43\leq x_{3}\leq 0.47;0.49\leq x_{4}\leq 0.52;0.47\leq x_{5}\leq 0.52\\ 0.54\leq x_{6}\leq 0.56;0\leq y_{1}\leq 0.74;0\leq y_{2}\leq 0.59\text{.} \end{array}$$

The optimization model will be built based on the data in Table 5, and it is shown as follows:

(24) $$\begin{array}{c} Mo\;de\;l\;4\text{:}\\ \min\xi_{2}=d_{12}^{+}+d_{12}^{-}+d_{13}^{+}+d_{13}^{-}+d_{14}^{+}+d_{14}^{-}+d_{23}^{+}+d_{23}^{-}+d_{24}^{+}+d_{24}^{-}+d_{34}^{+}+d_{34}^{-}\\ s.t.\left\{\begin{array}{c} In\omega_{1}-In\omega_{2}+0.5-\left(0.3384+0.26\times x_{1}\right)-d_{12}^{+}+d_{12}^{-}=0\\ In\omega_{1}-In\omega_{3}+0.5-\left(0.3922+0.26\times x_{2}-0.06\times y_{1}\right)-d_{13}^{+}+d_{13}^{-}=0\\ In\omega_{1}-In\omega_{4}+0.5-\left(0.46\times x_{3}+0.54\times x_{4}\right)-d_{14}^{+}+d_{14}^{-}=0\\ In\omega_{2}-In\omega_{3}+0.5-\left(0.3272+0.31\times x_{5}\right)-d_{23}^{+}+d_{23}^{-}=0\\ In\omega_{2}-In\omega_{4}+0.5-0.4598-d_{24}^{+}+d_{24}^{-}=0\\ In\omega_{3}-In\omega_{4}+0.5-\left(0.3127+0.41\times x_{6}-0.02\times y_{2}\right)-d_{34}^{+}+d_{34}^{-}=0\\ \overset{4}{\underset{r=1}{\sum }}\omega_{i}=1\\ 0\leq \omega_{i}\leq 1\;\\ 0\leq d_{jk}\leq 1\;\\ 0.50\leq x_{1}\leq 0.54\\ 0.48\leq x_{2}\leq 0.52\\ 0.43\leq x_{3}\leq 0.47\\ 0.49\leq x_{4}\leq 0.52\\ 0.47\leq x_{5}\leq 0.52\\ 0.54\leq x_{6}\leq 0.56\\ 0\leq y_{1}\leq 0.74\\ 0\leq y_{2}\leq 0.59\\ i,j,k=1,2,3,4 \end{array}\right.\text{.} \end{array}$$

The above model can be solved with the help of the Lingo software, and the results are shown as follows:

(25) $$\begin{array}{c} \xi_{2}=0.0563\text{,}\\ \omega_{1}=0.2444283;\omega_{2}=0.2485094;\omega_{3}=0.2553364;\omega_{4}=0.2517258\text{,}\\ x_{1}=0.54;x_{2}=0.48;x_{3}=0.4374795;x_{4}=0.4987803;x_{5}=0.47;x_{6}=0.54\text{;} \end{array}$$

(26) $$\begin{array}{c} y_{1}=0.74;y_{2}=0.59\text{;}\\ d_{12}^{+}=0.004640146;d_{23}^{-}=0.01625985;d_{24}^{+}=0.02734181;d_{34}^{-}=0.008058187\text{,}\\ d_{12}^{-}=d_{13}^{+}=d_{13}^{-}=d_{14}^{+}=d_{14}^{-}=d_{23}^{+}=d_{24}^{-}=d_{34}^{+}=0\text{.} \end{array}$$

We can find that all unknowns can be obtained by solving the above model; moreover, the value of the consistency degree *CI*_2_ can be calculated according to equation (8); the value is *CI*_2_=0.00938 after calculation, and the inequality *CI*_2_ < Ω holds which indicates that the results have met the consistency requirement; therefore, the adjustment module does not need to be activated, and the result is *A*_3_≻*A*_4_≻*A*_2_≻*A*_1_ according to the innovative ability.

### 4.4. The Comparison Algorithm with Related Unknowns

In this category, the data also contain several unknowns; moreover, different from the previous case, some unknowns are related to each other, and unknowns are not completely independent, such as the data in Table 6.


(27) $$\begin{array}{c} 0.50\leq x_{1}\leq 0.54;x_{2}=x_{1}+0.2;x_{3}=1.2\times x_{1};0.28\leq y_{1}\leq 0.35;y_{2}+y_{3}+y_{4}=1;0.2\leq y2\leq 0.4\\ 0.3\leq y3\leq 0.45;0.35\leq y4\leq 0.57;0\leq x_{2}\leq 1;0\leq x_{3}\leq 1;0.51\leq x_{4}\leq 0.55;0.53\leq x_{5}\leq 0.56\\ 0.3\leq y_{5}\leq 0.38;y_{6}=y_{5}-0.1;0\leq y_{6}\leq 1\text{.} \end{array}$$

(28) $$\begin{array}{c} Mo\;de\;l\;5\text{:}\\ \min\xi_{3}=d_{12}^{+}+d_{12}^{-}+d_{13}^{+}+d_{13}^{-}+d_{14}^{+}+d_{14}^{-}+d_{23}^{+}+d_{23}^{-}+d_{24}^{+}+d_{24}^{-}+d_{34}^{+}+d_{34}^{-}\\ s.t.\left\{\begin{array}{c} In\omega_{1}-In\omega_{2}+0.5-\left(0.344+0.29\times x_{1}\right)-d_{12}^{+}+d_{12}^{-}=0\\ In\omega_{1}-In\omega_{3}+0.5-\left(0.37+0.26\times x_{2}-0.02\times y_{1}\right)-d_{13}^{+}+d_{13}^{-}=0\\ In\omega_{1}-In\omega_{4}+0.5-0.5206-d_{14}^{+}+d_{14}^{-}=0\\ In\omega_{2}-In\omega_{3}+0.5-\left(0.48\times y_{2}{+x}_{3}\times y_{3}+0.52\times y_{4}\right)-d_{23}^{+}+d_{23}^{-}=0\\ In\omega_{2}-In\omega_{4}+0.5-0.512-d_{24}^{+}+d_{24}^{-}=0\\ In\omega_{3}-In\omega_{4}+0.5-\left(x_{4}\times y_{5}+0.55\times y_{6}{+x}_{5}-x_{5}\times y_{5}-x_{5}\times y_{6}\right)-d_{34}^{+}+d_{34}^{-}=0\\ \overset{4}{\underset{r=1}{\sum }}\omega_{i}=1\\ 0\leq \omega_{i}\leq 1\;\\ 0\leq d_{jk}\leq 1\;\\ 0.50\leq x_{1}\leq 0.54\\ x_{2}=x_{1}+0.2\\ 0.28\leq y_{1}\leq 0.35\\ y_{2}+y_{3}+y_{4}=1\\ 0.2\leq y_{2}\leq 0.4\\ 0.3\leq y_{3}\leq 0.45\\ 0.35\leq y_{4}\leq 0.57\\ x_{3}=1.2\times x_{1}\\ 0.51\leq x_{4}\leq 0.55\\ 0.53\leq x_{5}\leq 0.56\\ 0.3\leq y_{5}\leq 0.38\\ y_{6}=y_{5}-0.1\\ i,j,k=1,2,3,4 \end{array}\right.\text{.} \end{array}$$

The above model can be solved with the help of the lingo software, and the results are shown as follows:

(29) $$\begin{array}{c} \xi_{3}=0.0708\\ \omega_{1}=0.2543168;\omega_{2}=0.2541642;\omega_{3}=0.2423875;\omega_{4}=0.2491315\\ x_{1}=0.54;x_{2}=0.74;x_{3}=0.648;x_{4}=0.51;x_{5}=0.53\text{;} \end{array}$$

(30) $$\begin{array}{c} y_{1}=0.35;y_{2}=0.2739702;y_{3}=0.3;y_{4}=0.4260298;y_{5}=0.3;y_{6}=0.2\\ d_{13}^{-}=0.007358808;d_{24}^{+}=0.008;d_{34}^{-}=0.05544119\\ d_{12}^{+}=d_{12}^{-}=d_{13}^{+}=d_{14}^{+}=d_{14}^{-}=d_{23}^{+}=d_{23}^{-}=d_{24}^{-}=d_{34}^{+}=0\text{.} \end{array}$$

All unknowns can be obtained by solving the above model and all constraints are satisfied; moreover, the value of the consistency degree *CI*_3_ can be calculated according to equation (8), the value is *CI*_3_=0.0118 after calculation, and the inequality *CI*_3_ < Ω holds which indicates that the results have met the consistency requirement; therefore, the adjustment module does not need to be activated; the result is *A*_1_≻*A*_2_≻*A*_4_≻*A*_3_ according to the innovative ability.

## 5. The Comparisons and Discussion

Several data structures and processing methods proposed by other outstanding scholars will be compared with the data structure and algorithm proposed in the paper in this section.

### 5.1. The Probabilistic Linguistic Fuzzy Set and Its Processing Methods

The definition of the probabilistic linguistic fuzzy set is shown as follows:

(31) $$\begin{array}{c} L_{ij}=\left\{L_{l}\left(p_{l}\right)|L_{l}\in S,0\leq p_{l}\leq 1,l=1,2,\cdots ,k,\overset{k}{\underset{l=1}{\sum }}p_{l}=1\right\}. \end{array}$$

The symbol *L*_*l*_ represents the evaluation value, the symbol *p*_*l*_ represents its corresponding probability, the symbol *S* is called the additive linguistic set which contains all the possible evaluation values, the specific form is *S*={*s*_*a*_*|a*=0,1, ⋯, 2*τ*}, the symbol *τ* indicates an integer, the constraint condition *L*_*l*_ ∈ *S* indicates that all the evaluation values are from the additive linguistic set, the constraint condition 0 ≤ *p*_*l*_ ≤ 1 gives the value range of the probability, the symbol *k* indicates the total number of elements, and the constraint ∑_*l*=1_^*k*^*p*_*l*_=1 indicates that the sum of all the probabilities in a set must be equal to 1 [29].

Let us give a simple example to illustrate the above definition. Supposing the additive linguistic set is *S*={*s*_*a*_*|a*=0,1,2,3,4}, the symbol *s*_0_ indicates “terrible,” the symbol *s*_1_ indicates “bad,” the symbol *s*_2_ indicates “moderate,” the symbol *s*_3_ indicates “good,” and the symbol *s*_4_ indicates “excellent.” One of the typical probabilistic linguistic fuzzy sets can be denoted as *L*_12_={*s*_1_(0.45), *s*_2_(0.37), *s*_3_(0.18)}.

We can find that there are certain similarities with the definition of the incompletely probabilistic fuzzy set proposed in the paper. However, there are also differences between them, the main difference is the total number of the possible evaluation values, specifically, the number of possible evaluations in the probabilistic linguistic fuzzy set is limited; while, the number of possible evaluations in the incompletely probabilistic fuzzy set is infinite; in addition, the processing methods of incomplete information are not mature enough, and the data structure of probabilistic linguistic fuzzy set cannot contain multiple unknowns. These defects will seriously reduce the algorithm's accuracy.

### 5.2. The Probabilistic Hesitation Fuzzy Set and Its Processing Methods

Although the mathematical model of the probabilistic hesitation fuzzy set and the probabilistic linguistic fuzzy set has some similarities, there are still differences between them. Comparatively speaking, the probabilistic hesitation fuzzy set has more advantages in data processing, the operation rules, and the decision-making model, while the probabilistic linguistic fuzzy set can use linguistic terms to describe the real ideas of decision makers.

The probabilistic hesitation fuzzy set is an extension of the hesitation fuzzy set; its basic element is composed of the evaluation value and the corresponding probability [30]. In the decision-making process, the preference information given by experts can be described more comprehensively, and the uncertainty of a variety of possible scenarios can be simulated [31]. The definition of the probabilistic hesitation fuzzy set can be mathematically described as follows:

(32) $$\begin{array}{c} h_{r}=\left\{\gamma_{i}|p_{i}\;0\leq \gamma_{i}\leq 1,0\leq p_{i}\leq 1,\overset{k}{\underset{i=1}{\sum }}p_{i}=1,i=1,2,\cdots ,k\right\}. \end{array}$$

Supposing that there are two probabilistic hesitation fuzzy sets which can be denoted as *h*_1_={*γ*_*i*_*|p*_*i*_ *i*=1,2, ⋯, *k*_1_} and *h*_2_={*γ*_*j*_*|p*_*j*_ *j*=1,2, ⋯, *k*_2_}, respectively, the symbol *λ* indicates a positive real number. The basic rules of the probabilistic hesitation fuzzy set are listed as follows:

1. ${\left(h_{1}\right)}^{\lambda }=\underset{\gamma_{i}\in h_{1},p_{i}\in h_{1}}{\cup }\left\{\gamma_{i}^{\lambda }|p_{i}\right\}$
2. $\lambda h_{1}=\underset{\gamma_{i}\in h_{1},p_{i}\in h_{1}}{\cup }\left\{1-{\left(1-\gamma_{i}\right)}^{\lambda }|p_{i}\right\}$
3. $h_{1}⊕h_{2}=U\left\{\gamma_{i}+\gamma_{j}-\gamma_{i}\gamma_{j}|p_{i}p_{j}\right\}\begin{array}{c} \gamma_{i}\in h_{1},p_{i}\in h_{1}\\ \gamma_{j}\in h_{2},p_{j}\in h_{2} \end{array}$
4. $h_{1}⊗h_{2}=U\left\{\gamma_{i}\gamma_{j}|p_{i}p_{j}\right\}\begin{array}{c} \gamma_{i}\in h_{1},p_{i}\in h_{1}\\ \gamma_{j}\in h_{2},p_{j}\in h_{2} \end{array}$

The incompletely probabilistic fuzzy set proposed in the paper is extended from the probabilistic hesitation fuzzy set [32]. It inherits the advantages of the probabilistic hesitation fuzzy set, including basic calculation methods and theoretical models; on this basis, the incompletely probabilistic fuzzy set allows some unknowns to be included and the processing scope has been further expanded.

## 6. Conclusions

It is widely known that a scientific and reasonable evaluation mechanism is very important to promote the cultivation of students' innovative abilities [33]. The main purpose of this paper is to establish a high-discrimination evaluation mechanism of innovative ability. The innovative ability is a fuzzy definition and difficult to be measured by common algorithms.

At present, the common methods of dealing with this problem can be simply summarized as follows: several key indicators should be selected and these indicators will be scored separately; then, the scores will be aggregated by simple algebraic operation methods, and the aggregated value represents the innovation ability of the tested student. The above method is simple and efficient, but there are also some serious shortcomings. The value of each indicator is a single real-value, and it may be difficult to fully describe the details of the indicator [34]. The information aggregation method are too simple, and it is difficult to make full use of the indicator data [35].

After the above analysis, the paper combines the problem with fuzzy mathematics and tries to propose a new way to solve this problem. The data structure of the incompletely probabilistic fuzzy set proposed in the paper is developed from several definitions of fuzzy mathematics; it can save all possible values in a single dataset which can fully consider the hesitation and fuzziness in the process of data collection; and it also can fully accommodate different opinions of multiple experts. In addition, the incompletely probabilistic fuzzy set also allows unknowns to be included which enables more data details can be saved together. Compared with traditional methods, the pairwise comparison method is also one of the improvements; obviously, it is easier to obtain scientific and reasonable results by the pairwise comparison of alternatives. Since experts mainly focus on the work of pairwise comparisons, there may be contradictions among the comparison results from the overall perspective. To solve this problem, the definition of the consistency degree is proposed in the paper; moreover, the consistency optimization model is designed to estimate the values of the unknowns. The consistency degree can be obtained through the accumulation of deviation values. The automatic adjustment module will be activated if the consistency degree exceeds the warning threshold; this mechanism is also one of the innovations; it can improve the efficiency of the algorithm and accelerate the achievement of the consistency goal. After the above steps, the ranking of alternatives can be obtained according to the checked comparison data.

In order to verify the superiority of the algorithm, various experiments have been carried out; all the results have proved the effectiveness of the algorithm proposed in the paper, and then, several outstanding algorithms have been compared with the algorithm proposed in the paper; the results show that the algorithm proposed in this paper does have some advantages for solving this problem.

Honestly, although the algorithm is efficient, but it has not been fully verified in large projects, the algorithm with a feedback mechanism will be the research object of our team in the near future.

## Figures and Tables

**Figure 1:** The flowchart of the high-discrimination comparison algorithm.

**Figure 2:** The flowchart of the consistency automatic adjustment algorithm.

**Table 1:** The overall structure of the original data needs to be collected.

Indicators alternatives	*I*_1_	*I*_2_	⋯	*I*_*t*_
*A*_1_	*l*_11_	*l*_12_	⋯	*l*_1*t*_
*A*_2_	*l*_21_	*l*_22_	⋯	*l*_2*t*_
⋮	⋮	⋮	⋮	⋮
*A*_*m*_	*l*_*m*1_	*l*_*m*2_	⋯	*l*_*mt*_

**Table 2:** The structure of the comparison table.

Alternatives	*A*_1_	*A*_2_	⋯	*A*_*m*_
*A*_1_	*l*_11_	*l*_12_	⋯	*l*_1*m*_
*A*_2_	*l*_21_	*l*_22_	⋯	*l*_2*m*_
⋮	⋮	⋮	⋮	⋮
*A*_*m*_	*l*_*m*1_	*l*_*m*2_	⋯	*l*_*mm*_

**Table 3:** The simplified data structure of the comparison table.

Alternatives	*A*_1_	*A*_2_	⋯	*A*_*m*_
*A*_1_	{0.5*|*1}	*l*_12_	⋯	*l*_1*m*_
*A*_2_	1 − *l*_12_	{0.5*|*1}	⋯	*l*_2*m*_
⋮	⋮	⋮	⋮	⋮
*A*_*m*_	1 − *l*_1*m*_	1 − *l*_2*m*_	⋯	{0.5*|*1}

**Table 4:** The comparison data with complete information.

	*A*_1_	*A*_2_	*A*_3_	*A*_4_
*A*_1_	{0.5*|*1}	$\left(\begin{array}{c} 0.45\left|0.36,0.47\right|0.18\\ 0.49\left|0.24,0.52\right|0.22 \end{array}\right)$	$\left(\begin{array}{c} 0.46\left|0.32,0.49\right|0.23\\ 0.51|0.45 \end{array}\right)$	$\left(\begin{array}{c} 0.51\left|0.23,0.54\right|0.41\\ 0.56\left|0.22,0.58\right|0.14 \end{array}\right)$

*A*_2_		{0.5*|*1}	$\left(\begin{array}{c} 0.51\left|0.35,0.53\right|0.36\\ 0.55|0.29 \end{array}\right)$	$\left(\begin{array}{c} 0.46\left|0.44,0.48\right|0.25\\ 0.49|0.31 \end{array}\right)$

*A*_3_			{0.5*|*1}	$\left(\begin{array}{c} 0.52\left|0.35,0.54\right|0.51\\ 0.55\left|0.08,0.57\right|0.06 \end{array}\right)$

*A*_4_				{0.5*|*1}

**Table 5:** The comparison data with unrelated unknowns.

	*A*_1_	*A*_2_	*A*_3_	*A*_4_
*A*_1_	{0.5*|*1}	$\left(\begin{array}{c} 0.44\left|0.31,0.46\right|0.22\\ 0.48\left|0.21,x_{1}\right|0.26 \end{array}\right)$	$\left(\begin{array}{c} 0.47\left|y_{1},x_{2}\right|0.26\\ 0.53|0.74-y_{1} \end{array}\right)$	(*x*_3_|0.46, *x*_4_|0.54)
*A*_2_		{0.5*|*1}	$\left(\begin{array}{c} 0.46\left|0.55,x_{5}\right|0.31\\ 0.53|0.14 \end{array}\right)$	$\left(\begin{array}{c} 0.42\left|0.24,0.45\right|0.27\\ 0.47\left|0.31,0.51\right|0.18 \end{array}\right)$
*A*_3_			{0.5*|*1}	$\left(\begin{array}{c} 0.51\left|y_{2},x_{6}\right|0.41\\ 0.53|0.59-y_{2} \end{array}\right)$
*A*_4_				{0.5*|*1}

**Table 6:** The comparison data with related unknowns.

	*A*_1_	*A*_2_	*A*_3_	*A*_4_
*A*_1_	{0.5*|*1}	$\left(\begin{array}{c} 0.48\left|0.39,0.49\right|0.32\\ x_{1}|0.29 \end{array}\right)$	$\left(\begin{array}{c} 0.48\left|y_{1},x_{2}\right|0.26\\ 0.50|0.74-y_{1} \end{array}\right)$	(0.51|0.47,0.53|0.53)

*A*_2_		{0.5*|*1}	$\left(\begin{array}{c} 0.48\left|y_{2},x_{3}\right|y_{3}\\ 0.52|y_{4} \end{array}\right)$	$\left(\begin{array}{c} 0.49\left|0.37,0.52\right|0.32\\ 0.53|0.31 \end{array}\right)$

*A*_3_			{0.5*|*1}	$\left(\begin{array}{c} x_{4}\left|y_{5};0.55\right|y_{6}\\ x_{5}|1-y_{5}-y_{6} \end{array}\right)$

*A*_4_				{0.5*|*1}

## Data Availability

The data used to support the findings of this study are included whthin the paper and are obtained through practical investigations by our team.
